# Severe myocardial depression in a patient with aluminium phosphide poisoning: A clinical, electrocardiographical and histopathological correlation

**DOI:** 10.4103/0972-5229.53117

**Published:** 2009

**Authors:** Viral Shah, Seema Baxi, Tanmay Vyas

**Affiliations:** **From:** Department of Medicine, Government Medical College, Bhavnagar, Gujarat, India; 1 Department of Pathology, Government Medical College, Bhavnagar, Gujarat, India

**Keywords:** Aluminium phosphide, myocardial depression, myocyte vacuolation, myocytolysis, phosphide poisoning

## Abstract

Aluminium phosphide poisoning is very common in India. It is one of the most fatal poisons. The clinical spectrum of poisoning varies depending upon the dosage and duration of consumption. The main effect of the poison is due to the release of phosphine which inhibits cytochrome oxidase and thereby hampers cellular oxygen utilization. Almost any organ can be affected by aluminium phosphide poisoning. We report a case where the heart was the predominantly affected organ. We describe the clinical symptoms and signs and their correlation with electrocardiographic and histopathological examinations.

## Introduction

Aluminium phosphide (ALP) poisoning (Celphos) has emerged as a common cause of accidental poisoning in children with a mortality ranging from 37–100%.[1] Since ALP is commonly used as a fungicide and rodenticide in India, many reports of accidental poisoning with severe consequences have been noted both in adults and children. However, only a few cases from outside India have been reported. The spectrum of symptoms and signs and their severity depends upon the time lag between ALP ingestion and hospitalisation. The most common presentation is shock with cold and clammy skin, a weak thready pulse and severe hypotension often refractory to vasopressors. Arrhythmias are common in ALP poisoning and are attributed to various causes including hypomagnesemia. Neurological, gastrointestinal and renal involvement is also common and documented in many case reports. Myocardial depression is also reported in many cases. We report a case of ALP poisoning with severe myocardial depression. Serial ECGs and all cardiac events were recorded. A post mortem examination was conducted, with a special interest in the heart to record cardiac myocyte changes on biopsy.

## Case Report

A 40-year-old male patient came to the hospital with a history of ingestion of ALP with a suicidal intent (one tablet of Celphos - 3 gm). The time between consumption and hospital arrival was approximately 3 hours. On arrival the patient complained of epigastric pain and had tried to vomit three to four times in an attempt to remove the tablets. He was conscious and oriented, and looked very unwell. His pulse rate was 110 beats/minute and his blood pressure was 70/30 mmHg. Examination of the respiratory system was unremarkable. Cardivascularly he was in shock. The oxygen saturation was 90% with pulse oximetry at atmospheric temperature and air. We began aggressively resuscitating the patient. Two peripheral lines for resuscitation were inserted and gastric lavage conducted with saline. Vasopressor norepinephrine was administered as per the standard dosage and one liter of normal saline was infused within one hour. On the first day, investigations showed a HG of 12 gm%, total white cell count of 7000/cumm and a normal ABG. Serum total calcium was 9.2 mg/dl, serum magnesium was 2.33 mg/dl, serum sodium 143 meq/L, serum potassium 5.3 meq/L and serum bicarbonate was 20 mmol/L. Blood urea, serum creatinine and LFTs were normal. After two hours of gastric lavage we gave coconut oil through Ryle's tube. ECG recorded on arrival showed a broad QRS complex with ST elevation in mainly the inferior oriented leads mimicking inferior wall myocardial infarction [Figure 1]. Serum CPKMB was very high (290 U/L).

**Figure 1:** Showing ST elevation in inferior oriented leads mimicking inferior wall myocardial infraction

Over the next few hours the patient's blood pressure continued to fall despite being on maximum doses of norepinephrine infusion, we therefore started the patient on a dopamine infusion as per standard recommended doses. Over the next six hours of aggressive supportive measures, the patient continued to deteriorate. An ECG six hours after admission resembled myocardial infarction or pericarditis [Figure 2]. Electrolytes after six hours were normal except for a mild decrease in serum magnesium and hence, we started IV Magnesium therapy in the recommended dosage. On day 2, the patient was drowsy and could not maintain his saturation (80% saturation with oxygen) and therefore, the patient was intubated and ventilatory support was initiated. Blood pressure on the 2^nd^ day was 70/30 mm Hg and did not improve despite the maximum dose of dopamine and norepinephrine. ECG on the 2^nd^ day was suggestive of severe myocardial injury. Electrolytes were normal except for serum magnesium which was 3 mg/dl. We therefore stopped the magnesium infusion. Despite 48 hours of maximal resuscitative measures, the patient died. We conducted a post mortem examination. On autopsy the heart appeared to be normal on gross examination. The heart was removed for histopathological examination. Figures 3 and 4 show striking changes in the myocardial muscles. Histopathological findings showed that both the left and right ventricles as well as the interventricular septum were involved. Sections from both the apex and base of the heart showed changes. The right ventricle showed minimal changes and the interventricular septum was the worst affected. The changes comprised of areas of mild to severe myocyte vacuolation and areas of myoctyloysis and degeneration. There were areas of increased waviness of myocardial fibers.

**Figure 2:** Showing ST elevation with broad QRS complex mimicking anterior wall myocardial infarction with bundle branch block

**Figure 3:** Severe degree of vacuolation in myocytes. (H and E, ×40)

**Figure 4:** Necrosis and myocytolysis in many of the myocardial fibers. (H and E, ×40)

## Discussion

Aluminium phosphide (ALP) is used as a rodenticide and is a common agent used in suicide attempts in India. Most of the cases in India are reported from northern India.[2,3] Refractory myocardial depression from ALP toxicity is not uncommon and carries a mortality of up to 77% (37–100%).[1,4] Easy availability and no antidote makes it an ideal suicidal poison. Upon exposure to moisture, it liberates phosphine gas, which is absorbed rapidly by inhalation or through the cutaneous or enteral routes. Phosphine resembles cyanide in that it inhibits cytochrome oxidase and thereby hampers cellular oxygen utilization.[5]

The classical presentation of ALP is epigastric pain, nausea and cardiogenic shock reflected as severe refractory hypotension and is described in many case reports;[1–3,6,7] however, severe myocardial depression predominated in our case. There are a few case reports of survival in case of ALP poisoning when patients were treated with vegetable oils particularly with coconut oil and hence, we tried the same.[8,9]

Our patient had severe myocardial depression which could be correlated with serial ECG changes resembling myocardial infarction/ myocarditis or pericarditis. [Figure 1] in the initial hours resembles inferior wall myocardial infarction and later resembles extensive anterior wall myocardial infarction. We feel that the initially liberated phosphine may be absorbed through the stomach and diaphragm and affect the inferior wall first which rests on diaphragm and later the entire heart.(authors need to provide evidence of this mechanism being described before) ECG changes have been studied in detail in various studies[10–13] and include atrial fibrillation, supraventricular and ventricular tachycardia, ST-T changes, bundle branch blocks and AV conduction disturbances. We did not encounter any such ECG changes in our patient except ST-T changes and broad QRS complexes [Figures 1 and 2]. Broad QRS complex, ST-T changes along with raised cardiac marker CK-MB point to severe myocardial damage.

Controversies exist about the magnesium level and prognosis of poisoning.[14] There was no magnesium imbalance or any electrolyte disturbance seen in our patient though we administered magnesium to avoid hypomagnesemia induced arrhythmias and death.

As the heart was the predominant organ affected in our case, we studied the histology of the heart in detail to correlate the clinical and histological findings. Histopathological findings of myocyte vacuolation and myoctyloysis and degeneration are both suggestive of myocardial injury. The areas of increased waviness of myocardial fibers indicate an episode of myocardial infarction. Cellular infiltration as reported in some articles was minimal in our case and could be due to the fact that the full blown infarct occurred only some time before the patient succumbed.[15]

## References

[1] Chugh SN, Arora BB, Malhotra GC (1991). Incidence and outcome of aluminium phosphide poisoning in a hospital study. Indian J Med Res.

[2] Siwach SB, Yadav DR, Arora B, Dalal S, Jagdish (1989). Acute aluminium phosphide poisoning-an epidemiological clinical and histopathlogical study. J Assoc Phys India.

[3] Singh D, Jit I, Tyagi S (1999). Changing trends in acute poisoning in Chandigarh zone: A 25-year autopsy experience from a tertiary care hospital in northern India. Am J Forensic Med Pathol.

[4] Bogle RG, Theron P, Brooks P, Dargan PI, Redhead J (2006). Aluminium phosphide poisoning. Emerg Med J.

[5] Chefurka W, Kashi KP, Bond EJ (1976). The effect of phosphine on electron transport of mitochondria. Pesticide Biochem Physiol.

[6] Chugh SN, Ram S, Chugh K, Malhotra KC (1989). Spot diagnosis of aluminium phosphide ingestion: An application of a simple test. J Assoc Phys India.

[7] Singh S, Singh D, Wig N, Jit I, Sharma BK (1996). Aluminium phosphide poisoning: A clinico-pathologic study. J Toxicol Clin Toxicol.

[8] Shadnia S, Rahimi M, Pajoumand A, Rasouli MH, Abdollahi M (2005). Successful treatment of acute aluminium phosphide poisoning: Possible benefit of coconut oil. Hum Exp Toxicol.

[9] Goswami M, Bindal M, Sen P, Gupta SK, Avasthi R, Ram BK (1994). Fat and oil inhibit phosphine release from aluminium phosphide–its clinical implication. Indian J Exp Biol.

[10] Chugh SN, Juggal KL, Ram S, Singhal HR, Mahajan SK (1989). Hypomagnesemic atrial fibrillation in a case of aluminium phosphide poisoning. J Assoc Physic India.

[11] Raman R, Dulberg M (1985). Electrocardiographic changes in Quickphos poisoning. Indian Heart J.

[12] Chugh SN, Ram S, Singhal HR, Malhotra KC (1989). Significance of heart rate response in shock due to aluminium phosphide poisoning. J Assoc Phys India.

[13] Jain Sm, Bhami A, Sepaha GC, Sanghavi VC, Raman PG (1985). Electrocardiaograohic changes in aluminium phosphide poisoning. J Assoc Phys India.

[14] Siwach SB, Singh P, Ahlawat S, Dua A, Sharma D (1994). Serum and tissue magnesium content in patients of aluminium phosphide poisoning and critical evaluation of high dose magnesium sulphate therapy in reducing mortality. J Assoc Phys India.

[15] Tripathi SK, Gautam CS, Sharma PL (1992). Clinical pharmacology of aluminium phosphide poisoning. Indian J Pharmacol.

